RETRACTED

# Art Image Processing and Color Objective Evaluation Based on Multicolor Space Convolutional Neural Network

**DOI:** 10.1155/2021/4273963

**Published:** 2021-08-09

**Authors:** Liang Jing, Shifeng Lv

**Affiliations:** ^1^Hubei Institute of Fine Arts, Wuhan 430205, Hubei, China; ^2^Luxshare Precision Industry Co., Ltd., Shanghai 200126, China

## Abstract

A convolutional neural network's weight sharing feature can significantly reduce the cumbersome degree of the network structure and reduce the number of weights that need to be trained. The model can directly input the original image, without the process of feature extraction and data reconstruction in common classification algorithms. This kind of network structure has got a good performance in image processing and recognition. Based on the color objective evaluation method of the convolutional neural network, this paper proposes a convolutional neural network model based on multicolor space and builds a convolutional neural network based on VGGNet (Visual Geometry Group Net) in three different color spaces, namely, RGB (Red Green Blue), LAB (Luminosity *a b*), and HSV (Hue Saturation Value) color spaces. We carry out research on data input processing and model output selection and perform feature extraction and prediction of color images. After a model output selection judger, the prediction results of different color spaces are merged and the final prediction category is output. This article starts with the multidimensional correlation for visual art image processing and color objective evaluation. Considering the relationship between the evolution of artistic painting style and the color of artistic images, this article explores the characteristics of artistic image dimensions. In view of different factors, corresponding knowledge extraction strategies are designed to generate color label distribution, provide supplementary information of art history for input images, and train the model on a multitask learning framework. In this paper, experiments on multiple art painting data sets prove that this method is superior to single-color label classification methods.

## 1. Introduction

In deep learning, the convolutional network structure model is an algorithm with a high recognition rate. It has developed into a hot research field in many disciplines, especially in the research of digital image processing, image recognition, target tracking, etc. The original image avoids complicated preprocessing of the image and has the characteristics of hierarchical structure, few training parameters, and strong adaptability, so it has been widely used [1–3]. The weights on the plane are shared, so the number of parameters that the model needs to be trained is reduced, and the degree of the cumbersomeness of the model is also reduced [4]. Each convolutional layer in the network will be connected to the calculation layer used to extract image features again. This kind of special feature extraction method can not only effectively reduce the dimension of the extracted mapping plane but also has the characteristics of spatial invariance [5].

RETRACTED

Although the development time of digital image processing technology is relatively short, due to the wide application of computer technology, image processing and analysis have been paid attention to by people from all walks of life, gradually forming their own scientific system [6]. In the research and application of images, people are only interested in a certain part of the image or an area with special properties. The area that people are interested in is called the foreground of the image, and the other parts are called the background. Human recognition of color is composed of three indispensable parts: light, objects that can reflect light, human eyes, and the brain. The sensation produced by the light falling on the retina of the human eye forms color. Under the trigger of light, the human eye senses the three-color light to generate corresponding electrical signals [7–9]. The electrical signals are transmitted to the brain through the human nervous system, and finally, colors are produced in the brain. Through years of development, people's understanding of color has become deeper and deeper, and color has developed into a complex subject, which involves many subjects such as physics, biology, materials science, and even psychology [10]. It can be known from the process of color formation that color is a subjective feeling produced by the human brain on the color of an object. This feeling is difficult to describe with mathematical methods. Despite the unremitting efforts of people, after continuous research and demonstration, a large number of color theories, measurement techniques, and standards have been proposed [11].

This paper constructs a convolutional neural network model based on multiple color spaces. Some mainstream convolutional neural network classification models and application scenarios are introduced, and then a classification network based on VGGNet (Visual Geometry Group Net) is selected for model training. Specifically, the technical contributions of this article can be summarized as follows:

  First, this article proposes a multicolor space-based convolutional neural network model and conducts research from data selection and training, model building, etc. Converting a single-color label to a color label distribution does not increase the annotation information other than the style of the training sample, which also ensures that the research in this paper is fair when compared with other methods.
  Second, we use an end-to-end multitask learning framework to optimize the classification task of artistic painting style and the task of color label distribution at the same time. The color label distribution based on the dimensional information of art history enhances the ability to discriminate visual features during the training of the convolutional neural network.
  Third, through experiments on three art painting data sets, we prove that the proposed method can effectively use art history related information to assist the learning of visual features and improve the accuracy of art painting style classification. Compared with the latest art painting classification method, our method has obvious advantages in experimental results on different data sets.

RETRACTED

The rest of this article is organized as follows.  Section 2 discusses related work.  Section 3 analyzes the method and mechanism of artistic image color gamut mapping.  Section 4 builds a convolutional neural network model based on multiple color spaces. In Section 5, experiment comparison and result analysis are carried out.  Section 6 summarizes the full text.

## 2. Related Work

Related scholars have proposed a new parameter to improve the distinguishing ability of cognitive machines [12–14]. This parameter is a kind of inhibitory signal, which has the effect of restricting the activation of repetitive features by the node of the element. Many network models will remember certain feature-related content in the connection weight. According to Hebb's principle, a feature is repeatedly learned, and then it will be easier to find when it is classified later. There are also researchers who combine evolutionary computing principles with the theory of cognitive machines to weaken the learning of frequently occurring features [15]. The network can focus on other different features and improve the distinguishing performance. CNN can be regarded as an extension of the cognitive machine, and the cognitive machine can be used as a unique structure of CNN [16, 17].

Researchers have proposed a color migration algorithm between global images [18]. The algorithm transfers the color characteristics of one image to another image by using color space conversion and then using statistical analysis knowledge. In order to ensure the independence of each color channel, the algorithm is carried out in the CIELAB (International Commission on Illumination Luminosity *a b*) color space, and then a linear transformation of the image is determined, and the source image is transformed using the statistical characteristics of the image to ensure the result image [19]. Experimental results show that in images with strong color similarity, the algorithm can transfer the color characteristics of the target image to the source image and obtain satisfactory visual effects. If the similarity between the images is poor, it may even fail.

RETRACTED

Related scholars have applied higher-order moments to image color transfer [20]. The algorithm introduces the kurtosis and slope of high-order moments and then uses modulus transformation and power transformation to adjust the high-order moments such as kurtosis and slope of the source image data, which better preserves the details of the image. It is more similar to the distribution of the target image and achieves a good color migration effect. However, this algorithm has high time complexity and cannot be directly applied to occasions with high real-time requirements. Related scholars have proposed the idea of image multiresolution coloring [21]. When performing face coloring, the low-resolution part of the image is first colored, and then the high-resolution part of the image is color transformed. At the same time, the algorithm skips the colored blocks in the process of coloring gray pixels, so the coloring speed of the image is greatly improved. But the applicability of the algorithm is not very strong. Although it has a good effect on face coloring, the effect on other scenes is not very obvious. Later, some scholars put forward a brand-new idea of color harmony [22]. The algorithm uses a circular palette to transform the color of the image. At the same time, in order to make the image more real and natural, the algorithm also uses standard color templates to correct the result image, so that the result image has a good visual effect and makes the user look very comfortable and natural. But because this algorithm uses palette matching, it has strong subjective performance.

The interactive image segmentation method is to extract the part that people are interested in the target image for further analysis and processing. However, human vision is also subjective, and this subjectivity determines that people have subjective factors in determining the effect of image segmentation in the process of image segmentation. The human brain will comprehensively consider the image when performing image analysis, such as the overall layout of the image, the way it is composed, the basic tones, and the spatial relationship. Especially when faced with color images, the logical analysis ability of the human brain is difficult to achieve with traditional computer image segmentation technology [23]. The application of artificial intelligence technology to image segmentation is a very important research direction. Artificial intelligence technology has a wealth of prior knowledge through continuous “learning” so that when similar problems are encountered. The problem is dealt with, and the factor of the human visual system is added to the judgment of the image segmentation result, which can greatly approach the human visual discrimination system and effectively improve the effect of segmentation [24, 25]. All in all, human-computer interaction emphasizes the role of humans, so it can produce better results.

RETRACTED

## 3. Methods and Mechanisms of Color Gamut Mapping for Artistic Images

### 3.1. Color Gamut and Color Gamut Mapping

Color is represented by color space, which is also called a color model. It uses mathematical methods to visualize the color, making the color representation more intuitive, explaining the color in a way that people can understand and having a unified standard. For example, from the perspective of human eyes, colors can be defined by hue, saturation, and brightness according to human visual characteristics; in display devices, we use red, green, and blue phosphors to determine the amount of light. These amounts of light are used to describe colors in a mixed way. In terms of printing and printing equipment, people use the reflection and absorption of cyan, magenta, yellow, and black to produce the desired color. Essentially, the color space is expressed by a coordinate system and subspaces. A three-dimensional coordinate is usually used to describe the color space. Each point in the coordinate corresponds to a color. In the color gamut mapping process, the relationship between the main mapping objects and the mapping parameters involved is shown in Figure 1.

### 3.2. Description and Calculation of the Color Gamut Boundary

The partition maximization description method is to describe the color gamut boundary by recording the maximum radius in each subspace of the device-independent color space in the polar coordinate system. In each part of the color space, the color gamut of a group of colors is described by a matrix containing the largest extremum color, and the color gamut surface is generated based on this matrix. The calculation process is mainly divided into two parts, namely, calculating the color gamut boundary descriptor and calculating the intersection between the color gamut boundary and the mapping direction line.

The representation of the vertices of the partition can be in the form of chromaticity coordinates (*L*, *C*, *h*) or spherical coordinates (*z*, *θ*, PreLAB). The calculation of the spherical coordinate system is as follows:

(1) $$\begin{array}{c} z={\left[{\left(LE-L\right)}^{2}-{\left(aE-a\right)}^{2}-{\left(bE-b\right)}^{2}\right]}^{1/2},\\ \alpha =\arctan\left[\frac{\left(aE-a\right)}{\left(bE-b\right)}\right],\\ \theta =\arctan\left[\frac{\left(LE-L\right)}{{\left[\left|aE-a\right|-\left|bE-b\right|\right]}^{1/2}}\right]. \end{array}$$

Among them, *E* is the center point of the color gamut description, and the coordinates are (50, 0, 0), which can be determined by calculation or direct assignment. *r* is the distance from the color point to the center point, and *θ* is the in-plane angle when the hue angle is PreLAB, the range is 0°∼180°. According to PreLAB and brightness *L*^*∗*^ and hue angle *h*, the color space represented by the above spherical coordinate system is divided into *m∗n* partitions. The color gamut boundary described by this method is realized in the form of a matrix. The color points (PreLAB, *θ*, *z*) or (*L*^*∗*^, *C*^*∗*^, *h*) of the color gamut boundary of each partition are stored in the matrix. The accuracy of the description of the color gamut boundary is related to the number of partitions selected. We take the maximum coordinate value of the radius *r* in each partition to obtain the GBD matrix. If there is no color data point in a certain zone, it can be obtained by interpolation calculation of the closest GBD matrix data.

RETRACTED

For the entire GBD, *n* intersection points can be obtained. In addition, the intersection of the brightness axis and the plane determined by the GBD matrix is calculated. These points are the end points of the boundary of the linear color gamut. For its calculation, only the GBD matrix corresponding to the maximum or minimum value needs to be considered. The point with the maximum brightness value and the two adjacent points are formed into a triangle in turn, and then the intersection point of the triangle and the brightness axis is calculated. If the intersection point is within the triangle, the point is the boundary between the color gamut and the mapping direction line.

### 3.3. SGCK Color Gamut Mapping Mechanism

The algorithm first maps the lightness of the source image color to the lightness range of the target color gamut through the Sigmoidal function lookup table according to the chroma of the source image and then maps the chroma to the target color gamut by segmental compression in the iso-hue plane.

Map the colors in the source color gamut to the lightness dynamic range of the target device color gamut. The form of the sigmoid function is a one-dimensional lookup table obtained by the normal cumulative probability distribution function, and its mathematical expression is as follows:

(2) $$\begin{array}{c} S_{i}=\prod_{n=0}^{i-1}\frac{1}{\sqrt{2\pi }\sigma }\cdot e^{\left({\left(n/m-x_{0}\right)}^{2}\right)/\left(2\sigma \right)}. \end{array}$$

Among them, *i* represents the input value of the lookup table, *i* = 0, 1, 2,…, *m*, *m* ≥ 100, and *x*_0_ and *δ* are the average value and variance of the normal cumulative probability distribution, and its size is the same as that of the target color gamut. The minimum brightness *L∗r*min is related. *S*_*i*_ represents the output value of the corresponding lookup table when the input value is *i*. We transform the lookup table output *S* into the target color gamut:

(3) $$\begin{array}{c} S_{\text{LUT}}=\frac{\left[S_{i}-\min\left(S\right)\right]}{\max\left(S\right)-\min\left(S\right)}\cdot L*r\min-L*r\max. \end{array}$$

Among them, *L∗r*min and *L∗r*max represent the minimum lightness and maximum lightness of the target color gamut, respectively, and *S*_LUT_ represents the transformed lookup table output value.

RETRACTED

We map the chroma *C* corresponding to the lightness of the color in the source color gamut to the lightness range of the target color gamut, namely,

(4) $$\begin{array}{c} L*r=P_{C}\cdot L*s-P_{C}L*o. \end{array}$$

Among them,

(5) $$\begin{array}{c} P_{C}=1-{\left(\frac{\left|C\right|}{C+4*10^{4}}\right)}^{0.5}. \end{array}$$

*L∗r* represents the lightness after mapping.

### 3.4. Spatial-Domain Color Gamut Mapping Algorithm

It improves the mapping quality accordingly and can better preserve the spatial details in the source image. The colors in the source color gamut are mapped to the target color gamut one by one, and the relationship between the colors and the surrounding colors is not considered. Taking the HPMinΔ*E* algorithm as an example, the algorithm can be expressed as follows:

(6) $$\begin{array}{c} I\text{ out}=\text{Min}\Delta E\left(I\text{ in}\right)\cdot \text{HP}. \end{array}$$

Among them, *I*out is the mapped image and *I*in is the source image. The mapping process is shown in Figure 2.

Considering the spatial characteristics of the image, the colors in the source color gamut will be processed according to the relationship between them and the colors in the neighborhood. The spatial-domain adaptive mapping algorithm is optimized in terms of the preservation of saturation information and the preservation of the relationship between colors in the source area.

## 4. Convolutional Neural Network Model Based on Multicolor Space

### 4.1. Mainstream Feature Extraction Model

The algorithm based on `a convolutional neural network is to automatically extract image features through the network. From an algorithm perspective, the network structure of the convolutional neural network uses shared parameters, which can not only reduce the size of the memory required for operation but also reduce the number of training iterations. There is even no need to perform any preprocessing operations and feature extraction on the image in advance. Compared with other traditional algorithms, this is the advantage of the convolutional neural network algorithm. Through the analysis of the principle of the convolutional neural network, we can see that the “depth” of the network and the “size of the convolution kernel” are the key factors that affect the performance of the network model algorithm. Generally speaking, as the depth of the network deepens, the network's ability to characterize image features will become stronger; smaller convolutional checks will process images more refined, and there will be more RELU layers, and the network's ability to recognize images is stronger. According to the current development of the deep learning network structure, the depth and breadth of the network are constantly increasing, and most of the smaller convolution kernels are used. Inception-v3 network not only uses a smaller convolution kernel but also optimizes the network structure module.

RETRACTED

Since the texture features of natural images and computer images are essentially different, the texture features of the two can be extracted to identify NI images and CG images. Texture features are different from image features such as color and grayscale. Texture features are based on the statistical features of the image area, which can not only extract the surface structure and arrangement characteristics of the object but also will not fail due to local deviation. Texture features often have rotation invariance and have a certain resistance to noise, and LBP is the description operator that best reflects the texture of an image. We can see that MRELBP can describe the micro and macro texture features of the image, while CoALBP can describe the texture relationship between image blocks. Therefore, this paper chooses the MRELBP feature and improves on CoALBP to obtain the CCoALBP texture feature. Combining the two texture features, the source forensics of NI images and CG images are performed.

When it comes to deep convolutional neural networks, one has to mention several more classic convolutional neural network feature extraction models, namely AlexNet, VGGNet, GoogLeNet, and ResNet. They are very well trained on large-scale datasets such as ImageNet, which is excellent and has a strong ability to recognize and classify images in multiple categories. Therefore, this section first compares the performance of classic deep convolutional neural networks, compares their respective advantages and disadvantages, and then builds the deep convolutional neural network model of this article on this basis.

RETRACTED

The number of layers of AlexNet is relatively shallow, which is not suitable for the classification problem of this article; while the network level of GoogLeNet is similar to that of VGGNet, the size of its convolution kernel is not only 3 × 3 like VGGNet. In contrast, VGGNet is more suitable for this article; although the last ResNet performs better than VGGNet in Top-1 val.err, its network level is deeper and has the same convolution kernel size problem as GoogLeNet. With such a multilayer network structure, the number of layers has increased several times, but the performance has not increased several times. Therefore, when considering choosing a network, you need to balance the requirements and choose a suitable network structure.

Therefore, starting from reality, combined with the objective evaluation of colors in this article, VGGNet is more appropriate within the acceptable range of evaluation effect and accuracy.

### 4.2. Model Architecture Description

In view of the rich types of artistic images, the depth of the training network, and the unbalanced distribution of training samples, this paper proposes a convolutional neural network model based on multiple color spaces. The model architecture is shown in Figure 3.

The consideration is to select the feature extraction part of VGGNet, that is, the convolutional layer and the pooling layer. Therefore, in the training phase, the three-color space models will be trained separately and save the parameter weights. After space is extracted from the features of the convolutional neural network, it is connected to a model output selection determiner at the same time. This model output selection determiner will unify the detection results obtained by the three-color space models and output the final prediction result.

### 4.3. VGGNet Model

When building the network model of this article, this article chooses to build it based on VGGNet, but considering the actual problems of this article, there are still some changes when building it. The specific network structure is shown in Figure 4.

The VGGNet structure is shown in Figure 4. Compared to the original VGGNet-16, this article mainly modified the three fully connected layers, changing the two fully connected layers of 4096 to 2048 and the final fully connected layer of 1000.

The specific description of the model output judgment selector is shown in the following formula:

(7) $$\begin{array}{c} \text{Pre}=\left\{\begin{array}{c} \max\left(\text{PreRGB},\text{PreHSV}\right),\min\left(\text{PreRGB},\text{PreLAB}\right),\min\left(\text{PreHSV},\text{PreLAB}\right)\\ \max\left(\text{PreHSV},\text{PreLAB},\text{PreRGB}\right) \end{array}\right). \end{array}$$

Among them, Prediction is the final prediction category result, and PreRGB (Red Green Blue), PreHSV (Hue Saturation Value), PreLAB are the training prediction results in the three-color spaces of RGB, HSV, and LAB, respectively.

RETRACTED

The output of Prediction has two results; one is predicted with the highest confidence in the three-color spaces, namely Prediction1; the other is the second highest result, namely Prediction2. One of the two results is output as the main color, and one is output as the auxiliary color.

### 4.4. Sample Selection Strategy

The adopted multicolor space convolutional neural network structure corresponds to the same training and testing data set. We consider the problems in the problem description of this article: the increasing variety of artistic image colors, the troubles of deep learning training networks, and the unbalanced distribution of data samples in the training phase. Here is some processing in terms of training input data.

#### 4.4.1. Random Cross Distribution of Training and Test Sets

The distribution is shown in the following formula:

(8) $$\begin{array}{c} \gamma_{\text{RGB}}\cup \gamma_{\text{LAB}}\cup \gamma_{\text{HSV}}\;\subseteq \;\gamma ,\\ \gamma_{\text{RGB}}\cap \gamma_{\text{LAB}}\;⊄\;\Phi ,\\ \gamma_{\text{LAB}}\cap \gamma_{\text{HSV}}\;⊄\;\Phi ,\\ \gamma_{\text{RGB}}\cap \gamma_{\text{HSV}}\;⊄\;\Phi . \end{array}$$

#### 4.4.2. Random Image Reconstruction

After the data set is allocated, based on the characteristics of the data set in this article, select the position of the front hood of the car or the standard color image as the data set. The color value of the pixel is basically independent of the spatial position. When dividing the training set and test set, a random reconstruction strategy is adopted for the image. That is, half of all pixels of the image are randomly selected as the new image and used as the training and testing data set.

## 5. Experimental Comparison and Result Analysis

### 5.1. Discussion of Experimental Parameters

We discussed the hyperparameters involved in the experiment on the Painting91 style data set.  Figure 5 shows the experimental results of the hyperparameters PreRGB, PreHSV, and PreLAB under different parameter values, in which the value of the hyperparameter varies from 0 to 1.

We first study the influence of the change of the PreRGB value on the classification result. In order to achieve the best classification effect, we fix PreRGB to 0.8. Special attention is that after determining the values of hyperparameters PreHSV and PreLAB, we verified the value of PreRGB many times and confirmed the reliability and stability of PreRGB = 0.8.

RETRACTED

For the color label distribution of the place of origin, we set the color label corresponding to the actual style to 1, and set the other styles produced in the same place of origin to a fixed value. When the value of the hyperparameter PreHSV changes within a certain range (0.2–0.4), the classification accuracy is relatively stable. However, when the value of PreHSV is very small (for example, PreHSV = 0.1), the performance of using a color label distribution is similar to using a single-color label. On the contrary, when PreHSV is set to a larger value, the color label value corresponding to the actual style in the generated color label distribution is excessively cut. This is consistent with the downward trend in the classification results observed in the figure.

In this work, we fixed the hyperparameter PreHSV to 0.3 to obtain the best classification performance. We set the hyperparameter PreLAB in the art movement color label distribution to 0.3. We used different color label distributions and cross-validated the values of these hyperparameters on different data sets (fixed two of them and evaluated the other hyperparameter), and the experimental results were stable.

### 5.2. Analysis of the Results of the Single-Color Label Experimental Evaluation

For the art painting data set, the existing work usually only uses the actual color label to identify the style. Many studies have used the VGGNet model to obtain good classification performance in the task of recognizing artistic painting style.  Figure 6 shows the result of classification using a single-color label, which does not take into account the relevance of art history.

We fused the two origin time color label distributions, and the fused color label distribution obtained a better classification effect than the color label distribution using only one origin time generation strategy.

Figure 6 is the experimental result of generating the color label distribution based on a single art history related factor. In the distribution strategy, the time distance between some artistic styles appearing in adjacent orders is too large. For example, Renaissance style artworks prevailed from the fourteenth to sixteenth centuries. The time interval between the origins of the Renaissance and the Baroque style is more than 100 years. Even if we reduce the time distance through standardized operations, this is still too big. On the contrary, although the first generation strategy of origin time only considers the order in which artistic styles are generated, it can effectively avoid the imbalance in time distance between styles. The experimental results of the color label distribution on the Painting91 style data set generated by using the origin factor have been greatly improved, which means that the origin information can effectively reflect the development of artistic style. The artistic styles produced in the same place of origin under the same art history background will influence each other, so these styles have high similarities. There may be a certain degree of inheritance between styles in the same artistic movement period.

RETRACTED

### 5.3. Analysis of the Results of the Evaluation of the Multicolor Label Distribution Experiment

We first generate single-factor color label distributions according to four different color label distribution generation strategies (two origin time color label distributions, one origin color label distribution, and one art movement color label distribution). In the process of training, relevant information of art history is integrated, and the relationship between styles can be reflected in the color label distribution. By optimizing the classification loss and style distribution loss, the deep model can learn various connections between styles in the field of art history.

Figure 7 shows the experimental results of the proposed method and other art painting style classification methods. The method proposed in this paper obtains an average of 92.5% classification results on the Painting91 style data set.

In Figure 8, we show the time it takes to objectively evaluate colors on the Painting91 style data set. Among them, the time-consumed of traditional CNN is about 0.36 s on average, which is higher than the time-consumed of multicolor space CNN.

## 6. Conclusion

This paper proposes a multicolor space-based convolutional neural network model, which is trained in three different color spaces, namely RGB, LAB, and HSV color spaces, and chooses to use VGGNet for feature extraction and prediction of color images. The predicted category results of the three models are then passed through a model output selection judge to perform the top2 output of the model as the final predicted category. The article analyzes the network structure and each process in detail, obtains a specific algorithm description after discussion, and obtains the convolutional neural network model of this article. This paper proposes an artistic painting style learning framework for the distribution of color labels. The proposed color label distribution generation strategy is used to encode the collected three types of artistic background information, and a set of color label distributions are generated for each type of style instance to express the relationship between artistic styles. In the training process, the network uses the joint loss to optimize the artistic style classification task and the color label distribution task at the same time. By optimizing the color label distribution, the background knowledge of art history can be learned to assist in enhancing the accuracy of style classification. This paper verifies the effectiveness of this method on multiple art painting data sets and obtains a good classification effect. This idea of using color label distribution learning to provide nonvisual dimension related information for visual image classification tasks can also be extended to more research.

RETRACTED

However, there is no unified and standard method that can effectively evaluate the quality of various digital color images. In order to verify the effect of the algorithm proposed in this article, the data obtained from the designed objective and subjective evaluation experiments are only used for research and cannot be applied to the development of related products. In addition, it is necessary to further improve the color gamut mapping theory and mechanism and continuously improve its application effects. Due to the rapid development of spectrum-based high-fidelity color reproduction, spectrum-based color management systems have gradually entered the practical application stage. The development of multiprimary color imaging equipment should be combined with the development of spectral data-based color gamut mapping and method research.

## Figures and Tables

**Figure 1:** The main mapping objects and mapping parameters in color gamut mapping.

**Figure 2:** Schematic diagram of the influence of HPMinΔ*E* color gamut cropping algorithm on image quality after mapping.

**Figure 3:** Convolutional neural network model architecture based on multicolor space.

**Figure 4:** The VGGNet structure of this article.

**Figure 5:** Simulation of hyperparameters of convolutional neural network based on multicolor space. (a) Hyperparameter PreRGB simulation, (b) Hyperparameter PreHSV simulation, and (c) Hyperparameter PreLAB simulation.

**Figure 6:** The ablation experiment results of the art painting style learning framework based on the color label distribution on the Painting91 style data set.

**Figure 7:** Experimental results on the Painting91 style data set.

**Figure 8:** The time consumption of different methods on the Painting91 style data set.

## Data Availability

The data used to support the findings of this study are available from the corresponding author upon request.
